The article "Mining TCGA database for tumor mutation burden and their clinical significance in bladder cancer" was published in 2020. Journal: Biosci Rep.

# Mining TCGA database for tumor mutation burden and their clinical significance in bladder cancer

**DOI:** 10.1042/BSR20194337

**Published:** 2020-04-21

**Authors:** Jia Lv, Yongze Zhu, Alin Ji, Qi Zhang, Guodong Liao

**Affiliations:** 1 Department of Urology, Zhejiang Provincial Peoples’ Hospital, Peoples’ Hospital of Hangzhou Medical College, Hangzhou 310014, China; 2 Department of Laboratory, Zhejiang Provincial Peoples’ Hospital, Peoples’ Hospital of Hangzhou Medical College, Hangzhou 310014, China

**Keywords:** Bladder Cancer, Immune cell infiltration, TCGA, Tumor mutation burden

## Abstract

*Background:* Bladder cancer is the ninth most-common cancer worldwide and it is associated with high morbidity and mortality. Tumor mutational burden (TMB) is an emerging biomarker in cancer characterized by microsatellite instability. TMB has been described as a powerful predictor of tumor behavior and response to immunotherapy.

*Methods:* A total of 443 bladder cancer samples obtained from The Cancer Genome Atlas (TCGA) were analyzed for mutation types, TMB values, and prognostic value of TMB. Differentially expressed genes (DEGs) were identified from the TMB groupings. Functional analysis was performed to assess the prognostic value of the first 30 core genes. CIBERSORT algorithm was used to determine the correlation between the immune cells and TMB subtypes.

*Results:* Single nucleotide polymorphism (SNP) and C>T were reported as the most common missense mutations and we also identified a high rate of mutations in TP53, TTN, KMT2D. Bladder cancer patients with high TMB showed a better prognosis. Enrichment analysis of the DEGs revealed that they were involved in the regulation of the P13K-Akt signaling pathway, cytokine–cytokine receptor interaction, and Ras signaling pathway. The high expression of hub genes *ADRA2A, CXCL12, S1PR1, ADAMTS9, F13A1*, and *SPON1* was correlated with poor overall survival. Besides, significant differences in the composition of the immune cells of T cells CD8, T cells CD4 memory activated, NK cells resting and Mast cells resting were observed.

*Conclusions:* The present study provides a comprehensive and systematic analysis of the prediction of TMB in bladder cancer and its clinical significance. Also, the study provides additional prognostic information and opportunities for immunotherapy in bladder cancer.

## Introduction

Bladder cancer, the ninth most-common malignancy worldwide with an estimated 356000 new cases and 145000 deaths annually, has a propensity to relapse, requiring lifelong monitoring after diagnosis [1,2]. Until very recently, bladder cancer treatment had seen little progress since, over the last three decades, a limited range of treatment options with an overall 5-year survival rate was being used by clinicians to treat patients [3,4]. Approximately 25% of bladder cancer is muscle-invasive bladder cancer. Poor prognosis in muscle-invasive bladder cancer is reported with 85% of the patients dying within 2 years without treatment [5]. In recent years, the use of immunotherapy in the treatment of muscle-invasive and metastatic bladder cancer has shown great potential in clinical application [6]. However, there are no biomarkers for assessing the effectiveness of immunotherapy in bladder cancer.

The article "Mining TCGA database for tumor mutation burden and their clinical significance in bladder cancer" was published in 2020. Journal: Biosci Rep.

Tumor mutational burden (TMB) refers to the number of somatic mutations per 1 million bases, excluding single nucleotide polymorphism (SNP), germline, copy number variation, and structural variation [7,8]. TMB is an emerging characteristic of cancer and is associated with microsatellite instability [9,10]. TMB increase in the human cancer genome is attributed to endogenous factors and environmental damage [11]. Previous studies reveal that patients with high TMB have a significantly better response to immunotherapy [12]. Therefore, TMB is an emerging biomarker for the prediction of tumor behavior and response to immunotherapy [13].

The rapid development of next-generation sequencing (NGS) technology and the establishment of the Cancer Genome Atlas (TCGA, https://cancergenome.nih.gov) database has helped to generate many large-scale cancer genomic datasets and comprehensive bioinformatics analysis has been made possible. In the current study, gene expression profile data in bladder cancer were extracted from TCGA and the data used to investigate the potential function of TMB in immunotherapy and personalized/precision medicine decision-making.

## Methods

### Data download and analysis

TCGA is a cancer genomics program providing publicly available data that contributes to cutting-edge cancer studies (https://portal.gdc.cancer.gov). Gene expression profiles and associated clinicopathological data of bladder cancer patients were from the TCGA database on 1 August 2019. The samples included 414 cancer tissue samples and 19 adjacent tissue samples. The Masked Somatic Mutation data (varscan. Somatic. Maf) were obtained, analyzed, and visualized using the ‘maftools’ in R package [14].

### TMB value estimation

TMB is a measure of the total number of mutations per megabyte of tumor tissue. It is also the mutation density of tumor genes defined as the average number of mutations in the tumor genome including the total number of gene coding errors, base substitution insertions or deletions [15]. The 38 Mb is routinely taken based on the length of the human exon, so the TMB estimate for each sample is equal to the total mutation frequency/38. TMB per megabase is calculated by dividing the total number of mutations by the size of the coding region of the target.

The article "Mining TCGA database for tumor mutation burden and their clinical significance in bladder cancer" was published in 2020. Journal: Biosci Rep.

### Relationship between TMB value and overall survival

Kaplan–Meier analysis in R package was performed to investigate the prognostic value of TMB in bladder cancer.

### Relationship between TMB value and clinicopathological features

Analysis of the relationship between TMB values and clinicopathological features (age, gender, stage grading, tumor grade, and TMN staging) was performed in the R package.

### Identification of differentially expressed genes

Based on the median TMB value (5.132), the TMB group was divided into a high-TMB group and a low-TMB group. The ‘limma’ R package was utilized to identify TMB-related differentially expressed genes (DEGs) [16], and all DEGs with FDR <0.05 and |log2 FC| >0.5 were exported, and the ‘pheatmap’ R package used to perform hierarchical clustering.

### Functional analysis of DEGs

The gene ontology (GO) pathway enrichment analysis and KOBAS-Kyoto Encyclopedia of Genes and Genomes (KEGG) pathways analysis of DEGs were performed by ‘clusterProfiler, org.Hs.eg.db, plot, ggplot2’ in R package [17]. The protein–protein interaction (PPI) network of DEGs were constructed in the STRING database [18], and the number of core gene nodes in the PPI network were visualized using Cytoscape software in R package [19].

### Core gene survival analysis

The survival package in R was used to assess the prognostic value for the top 30 core genes in bladder cancer.

### CIBERSORT analysis

CIBERSORT is a deconvolution tool that uses linear support vector regression to determine the expression matrix of human leukocyte subtypes [20]. The abundance of 22 leukocyte subtypes in bladder cancer was obtained using the ‘CIBERSORT’ R package, with a cut-off *P*-value <0.05. Wilcox test was performed to analyze the differences not only in the immune cell abundance in the patients but also in the high-TMB and low-TMB groups which were visualized using the ‘beeswarm’ R package.

### Statistical analysis

R Studio v 1.1.463 and Bioconductor (https://www.bioconductor.org/) were used for statistical analysis [21]. Overall survival was assessed by Kaplan–Meier and log-rank test methods, and subgroup differences were analyzed by the Wilcox test or Kruskal test, with *P*-values <0.05 considered to be statistically significant.

## Results

### Mutations in bladder cancer

We first evaluated the variation in each TCGA bladder cancer sample to provide insights into the factors associated with bladder cancer mutagenesis. The findings revealed that missense mutations, SNP, and C>T mutation were more common, with the highest mutation frequency being 3398 (Figure 1A). Based on the MutSigCV algorithm, the waterfall diagram revealed the integration status of somatic mutations in TCGA bladder cancer, and the results showed that the somatic mutations of TP53, TTN, KMT2D, ARID1A, MUC16, PIK3CA, and RB1 (*P*<0.001) were higher (Figure 1B).

The article "Mining TCGA database for tumor mutation burden and their clinical significance in bladder cancer" was published in 2020. Journal: Biosci Rep.

**Figure 1:** TCGA bladder cancer mutation cohort (**A**) Overview of TGCA bladder cancer cohort mutations. (**B**) Waterfall of the top 30 mutated genes in the TCGA bladder cancer cohort.

### TMB and clinical relevance

Kaplan–Meier analysis was used to assess the potential correlation of TMB in bladder cancer with prognosis. The results showed that TMB (Figure 2A, *P*=0.004) was associated with prognosis. Patients with high-TMB had a better prognosis, suggesting that the patients experienced better effects on the immune response. The correlation between TMB and clinicopathological features including patients’ gender, tumor grade (tumor cell differentiation), and TNM staging revealed that TMB was associated with gender (Figure 2B, *P*=0.011) and tumor grade (tumor cell differentiation) (Figure 2C, *P*=3.663e-05) in patients with bladder cancer. The TMB of male patients was reported to be higher than that of female patients. Besides, bladder cancer patients with high tumor grade (well differentiation) had a higher TMB value.

**Figure 2:** TMB correlation analysis (**A**) Kaplan–Meier curves of overall survival of the high- and low-TMB groups. (**B**) Wilcox test for patients stratified by gender. (**C**) Wilcox test for patients stratified by grade.

### Enrichment analysis for the DEGs

TMB-associated DEGs in bladder cancer were analyzed using the ‘limma” package. A total of 506 DEGs were identified, including 181 up-regulated and 325 down-regulated genes. Figure 3 shows the hierarchical clustering heatmap. GO enrichment analysis was performed to elucidate the biological functions of the DEGs. Figure 4A shows the top 30 enriched GO terms which were associated with tumor immune cell response and composition of extracellular matrix (ECM). As shown in Figure 4B, KEGG pathway analysis showed that the DEGs were mainly enriched in the PI3K-Akt signaling pathway, cytokine–cytokine receptor interaction, Ras signaling pathway, chemokine signaling pathway, ECM–receptor interaction, and bladder cancer.

**Figure 3:** Hierarchical clustering heatmap of DEGs between high- and low-TMB groups The higher and lower expressed genes were shown in red and green, respectively, and genes with the same expression level in black.

**Figure 4:** Functional enrichment analysis of DEGs (**A**) Functional analysis of the top ten enriched biological processes (BPs), cell composition (CC), and molecular function (MF) of GO analysis. (**B**) KEGG enrichment diseases analysis.

The article "Mining TCGA database for tumor mutation burden and their clinical significance in bladder cancer" was published in 2020. Journal: Biosci Rep.

### PPI network of DEGs

The PPI network of the DEGs was constructed using the STRING online database to determine interactions among DEGs and discover important genes involved in tumorigenesis. The networks were visualized using the Cytoscape software (Figure 5A). Among the top 30 core genes with the highest clustering included *GNG4, GNG7, AGT, ADCY5, CXCL10, THBS1, ADRA2A* and *CXCL11* etc. (Figure 5B). Kaplan–Meier analysis was used to investigate the prognostic values of the 30 potential core genes (Figure 5B). In conclusion, high expression of ADRA2A (Figure 6A), CXCL12 (Figure 6B), S1PR1 (Figure 6C), ADAMTS9 (Figure 6D), F13A1 (Figure 6E), and SPON1 (Figure 6F) was associated with poor overall survival in bladder cancer patients, with a *P*-value <0.05 considered to be statistically significant.

**Figure 5:** PPI network analysis (**A**) PPI network. The color and size of the map node was determined by the degree value, which was a gradual process. Green and small circles represent low values, and orange and large circles represent high values. (**B**) Histogram of core genes.

**Figure 6:** The overall survival of bladder cancer patients with high or low expression of ADRA2D (**A**) CXCL12 (**B**) S1PR1 (**C**) ADAMTS9 (**D**) F13A1 (**E**) and SPON1(**F**).

### Association of TMB and tumor immune microenvironment

After the previous calculation, the proportion of 22 immune cells in all samples was obtained. The findings revealed that the first three sites in the low TMB group were macrophages M0 (0.155), macrophages M2 (0.1443), and T cells CD4 resting (0.1117), while in the high TMB group were T cells CD8 (0.1487), Macrophages M2 (0.1412), and Macrophages M0 (0.139), respectively (Figure 7). The differences in the abundance of each leukocyte subtype between the high- and low-TMB groups showed that samples with high-TMB had a significant increase in the abundance of T cells CD8 (*P*<0.001), T cells CD4 memory activated (*P*=0.002), and NK cells resting (*P*=0.023) and a significant decrease in the abundance of mast cells resting (*P*=0.011) (Figure 8). In conclusion, the difference in TIICs between the two groups suggests that they may have important clinical implications.

**Figure 7:** The average proportion of each type of tumor-infiltrating immune cells in in the low- and high-TMB groups

**Figure 8:** Differential analysis of tumor-infiltrating immune cells (TIICs) between high- and low-TMB groups

## Discussion

The tumorigenesis is a complex multistep process, involving genetic alterations interacting with immune cells in tumor microenvironment [22,23]. Somatic missense mutations strongly contribute to the generation of novel tumor epitopes [13]. A better understanding of the relationship between TMB with highly immunogenic tumors may help to evaluate the effect of immunotherapy and provide a mechanistic explanation for the observed clinical survival patterns. Immune checkpoint molecule inhibitors have opened the possibility of immunotherapy for bladder cancer, especially for muscle-invasive and metastatic bladder cancer [24,25]. Recent research has correlated bladder cancer and the immune environment [26]. However, there are no available biomarkers to assess the effectiveness of immunotherapy in bladder cancer.

The article "Mining TCGA database for tumor mutation burden and their clinical significance in bladder cancer" was published in 2020. Journal: Biosci Rep.

In the present tudy, we analyzed mutations in bladder cancer samples. The findings revealed that missense mutations, SNP, and C>T mutations were the most common mutation forms in bladder cancer. Previous studies have demonstrated the significance of missense mutation and SNP in tumorigenesis, progression, and prognosis in various cancer types, including bladder cancer [27–30]. The three most frequently mutated genes were *TP53, TTN*, and *KMT2D*. TP53 is one of the famous tumor suppressor genes reported to regulate the cell cycle thus inhibits the development of cancerous cells [31]. P53 protein maintains genome stability and prevents the occurrence of genomic mutation [32]. KMT2D is a known cancer-related protein that regulates tumor growth and metastasis, thus influences prognosis [33,34]. In bladder cancer, KMT2D functions as a tumor suppressor and supports tumor cell viability, migration, and invasion [35].

The clinical significance of TMB in bladder cancer was analyzed. The results showed that TMB was higher in bladder cancer patients with high tumor grade. Bladder cancer patients with low TMB had a poor prognosis compared with those with high TMB. These results demonstrated that high-TMB often has a relatively favorable living condition. In breast cancer, TMB is a determinant of immune-mediated survival of patients and identify candidate immune-regulatory mechanisms associated with immunologically cold tumors [36]. Therefore, TMB is suggested to be an independent predictor of immunotherapy response in various types of cancers including bladder cancer [37–39].

The potential biological functions of TMB-associated DEGs were analyzed. The functions of TMB-associated DEGs were mainly associated with tumor immune cell response, PI3K-Akt signaling pathway, cytokine–cytokine receptor interaction, Ras signaling pathway, chemokine signaling pathway, ECM–receptor interaction, and bladder cancer. The PI3K/AKT signaling pathway shows frequent molecular alterations and increased activity in cancers. Previous studies have revealed the significant role of the PI3K/AKT pathway in bladder cancer. Leupaxin promotes bladder cancer proliferation, metastasis, and angiogenesis through the PI3K/AKT pathway [40]. Another study revealed that activation of the PI3K/AKT pathway plays a critical role in the initiation and progression of bladder cancer [41,42]. Ras signaling pathway is considered to exert an important role in tumorigenesis and progression of human cancers, including RCC and bladder cancer [43,44]. The immense diversity of ECM proteins confers distinct biochemical and biophysical properties that influence cell phenotype. The composition and organization of the ECM are spatiotemporally regulated to control cell biological processes (BPs), but an aberrant expression of ECM dynamics results in the occurrence of diseases such as cancer [45].

The article "Mining TCGA database for tumor mutation burden and their clinical significance in bladder cancer" was published in 2020. Journal: Biosci Rep.

Kaplan–Meier analysis demonstrated the TMB-associated DEGs PPI network. *ADRA2A, CXCL12, S1PR1, ADAMTS9, F13A1*, and *SPON1* were selected as the hub genes which were reported to be mainly involved in DNA replication, cell cycle control, genomic stability, and mitosis [46–49]. Besides, the hub genes regulate tumor cell proliferation, invasion, apoptosis, and metastasis [50,51]. Therefore, the present study demonstrated that the identified hub genes played a significant role in bladder cancer.

The correlation between TMB and tumor-infiltrating immune cells was analyzed to reflect on the status of the immune microenvironment. In the current study, there was a significant increase in the abundance of T cells CD8, T cells CD4 memory activated, and NK cells resting and a significant decrease in the abundance of Mast cells resting in the high-TMB group compared with the low-TMB group. These results demonstrate that patients with higher infiltration levels of CD8^+^ T cell, CD4 T cell, NK resting cells, and lower Mast cells are more likely to present with better immunotherapeutic effect and prognosis. These findings confirm that CD4, CD8 T cells, and NK cells, may be major players in antitumor immunity in bladder cancers in patients with high TMB.

The presentstudy was not without limitations that should be considered when interpreting our results. For instance, the results of the current study were not validated using an independent patient cohort. Thus, further *in vitro* or *in vivo* experiments are needed to validate our findings.

## Conclusion

In conclusion, the present study provides a comprehensive and systematic analysis of the prediction of TMB in bladder cancer and its clinical significance in the recognition, surveillance, and prognosis of bladder cancer. In addition, the present study provides additional prognostic information and opportunities for immunotherapy in bladder cancer.

The article "Mining TCGA database for tumor mutation burden and their clinical significance in bladder cancer" was published in 2020. Journal: Biosci Rep.

## Abbreviations

DEG: differentially expressed gene
ECM: extracellular matrix
FDR: false discovery rate
GO: gene ontology
KEGG: Kyoto Encyclopedia of Genes and Genomes
KOBAS: KEGG Orthology Based Annotation System
NK: Natural killer
PPI: protein–protein interaction
RCC: Renal cell carcinoma
SNP: single nucleotide polymorphism
TCGA: The Cancer Genome Atlas
TMB: tumor mutational burden
TMN: Tumor, Node, Metastasis
